# Cloud-Based Fault Prediction Using IoT in Office Automation for Improvisation of Health of Employees

**DOI:** 10.1155/2021/8106467

**Published:** 2021-11-03

**Authors:** Mudita Uppal, Deepali Gupta, Sapna Juneja, Gaurav Dhiman, Sandeep Kautish

**Affiliations:** ^1^Chitkara University Institute of Engineering and Technology, Chitkara University, Punjab, India; ^2^IMS Engineering College, Ghaziabad, India; ^3^Government Bikram College of Commerce, Patiala, India; ^4^LBEF Campus, Kathmandu, Nepal

## Abstract

The novel paradigm of Internet of Things (IoT) is gaining recognition in the numerous scenarios promoting the pervasive presence of smart things around us through its application in various areas of society, which includes transportation, healthcare, industries, and agriculture. One more such application is in the smart office to monitor the health of devices via machine learning (ML) that makes the equipment more efficient by allowing real-time monitoring of their health. It guarantees indoor comfort as per the user's satisfaction as it emphasizes on fault prediction in real-life devices. Early identification of various types of faults in IoT devices is the key requirement in smart offices. IoT devices are becoming ubiquitous and provide an assistant to supervise an office that is regulated by ML and data received from sensors is stored in cloud. A recommender system facilitates the selection of an appropriate solution for faults in IoT-enabled devices to mitigate faults. The architecture proposed in this paper is used to monitor each and every office appliance connected via IoT technology using ML technique, and recommender system is used to recommend solutions for fault patterns without much human intervention. The ultrasonic motion sensor is used to fetch the information of employee availability in cubicles and data is sent to the cloud through the WiFi module. ATmega8 is used to control electrical appliances in the office environment. The significance of this work is to forecast the faults in IoT appliances which will have an impact on life and reliability of IoT appliances. The main objective is to design a prototype of a smart office using IoT that can control and automate workplace devices and forecast whether the device needs repairing or replacing, thus reducing the overall burden on the employee and helping out in increasing physical as well as mental health of the person.

## 1. Introduction

The 21^st^ century is witnessing a fast-paced digital revolution. Internet of Things (IoT) is a recent concept in which real-world physical entities can be remotely controlled with the help of the Internet. IoT architecture contains a physical object network that is integrated with sensors, electronic devices, and software which allow them to gather and transfer data through an IoT network. These entities are also called smart objects because they can sense the environment and can be remotely controlled through existing IoT network architecture by integrating with the physical environment. IoT has a positive impact on daily lives as it provides new solutions to every aspect of society. Therefore, IoT is a phenomenon that results in an event between the sensor, real-time network, and the data centres [1].

In an IoT application, the perception layer consists of smart objects embedded with sensors that collect and process real-time information of the physical and digital worlds. These sensors help in the measurement of the physical resources and monitor the changes in the physical environment [2].  Figure 1 represents the architecture of an IoT application [7].

There is a need for memory in the gateway to receive the sensor data that the sensors send to the gateways. Sometimes, these sensors generate a large amount of data that need a robust and high-performance WSN that transports these data to the destination gateway on time. Several protocols and technologies are needed in the heterogeneous configuration of an IoT application [8]. Also, a broad range of IoT services or applications like speed transactions, compatibility, or context-aware applications are demanded.

IoT is gaining popularity worldwide in different situations of the advanced wireless communications network while supporting the presence of smart things around us. IoT is capable of changing the world [9]. There has been an abundance of information and this advanced technology has opened many paths to access this information. Every part of our lives is getting changed by the development of IoT [10]. IoT frameworks are intensely used in many applications as demonstrated below.  Figure 2 outlines some of the fundamental areas and applications of IoT which includes smart traffic system, smart environment, smart healthcare, smart home, smart agriculture, smart office, and supply chains logistics IoT [14–16].

Smart office automation is the latest and upcoming technology in the market that is easier to control and makes life simpler. A smart office is a place where one would find desktop computers and printers connected to a router via cable for Internet access. Also, appliances like laptops, printers, smart heaters, smart window blinds, coffee machines, etc., are all connected to the Internet.

There are many advantages of IoT, but still there are some issues that must be addressed to advance its growth [17]. The applicability of IoT devices is a complex mixture of various technologies that provide solutions based on the integration of various heterogeneous technologies. In many cases, IoT applications heavily depend on a network of connected components embedded in physical objects, such as appliances or devices [18]. The functionality and operation of these physical objects are important in communication and connectivity. The complexity of these devices and technology leads to the challenge of creating a dependable IoT application [19].

Cloud computing uses central remote servers to manage data and applications via the Internet. It allows users to run applications without installing them or directly accessing their files at any time on any machine having Internet access. It provides on-demand computing services such as applications, storage, and processing power. Cloud gives several services to the client like Platform as a Service (PaaS), Software as a Service (SaaS), and Infrastructure as a Service (IaaS) [20]. The integration of cloud and IoT leads to the expansion of available technologies in cloud environments. The information and applications used by the IoT technology can be stored on cloud storage. The integration of cloud and IoT technology is represented in Figure 3. Cloud allows users to access all the information needed for IoT connectivity [24].

Energy is an important technological challenge in IoT and in-depth research is required to develop systems that can save energy during the operational environment [25, 26]. IoT needs ways to minimize the energy spent on communication and computing. Also, it requires techniques to harvest energy that will assist IoT devices to relieve from the restrictions foisted by battery operations, scarce energy, and limited resources that need to be tackled in IoT applications. Therefore, there is a need to devise solutions that will optimize energy usage in IoT devices [27]. Also, early fault prediction can extend equipment life, increase safety, and reduce manufacturing costs [28]. Fault prediction is a crucial aspect to be evaluated because it helps in determining the fault proneness of IoT devices. The elimination of faults enhances the quality and improves the effectiveness of the whole process. Machine Learning (ML) acts as a key factor in fault prediction and helps in getting more accurate results. ML has many techniques and algorithms, such as Artificial Neural Networks, Multilayer Perceptron, Naive Bayes, Genetic Algorithms, and many more that can be used in fault prediction and save time [29]. ML can automatically examine heterogeneous data by applying smart algorithms and models to achieve better results. The techniques and algorithms used in ML are different from one another in terms of their working, hypotheses, properties, precision, advantages, disadvantages, and solving category. The actions required to find the faulty devices are planned earlier in case of any problem. The consequences can be catastrophic if faults are not tackled beforehand and they may also disrupt the actual result [30, 31].

IoT is a booming shift in the IT epoch. IoT developments are accelerating innovation-driven information and technological applications in several areas such as production processes, agricultural fields and home or office automation. The increased demand for digital terminals configured with a robust variety of sensors enables a greater process of data acquisition module for industrial IoT. Prediction of faults is a big security challenge in IoT devices but still, it is one of the safe methods of fault prevention [32]. Smart automation has a significant impact on the customer's experience by giving fault-free solutions. Early prediction of faults plays a very important role in terms of quality measurement. ML-based approaches have been considered the most promising technique due to the learning mechanism of classifiers. To predict a fault before its occurrence reduces the overall cost and time and cost of the projects. Also, the need for a reliable and refined technique is a point of concern. IoT is a convergence of many technologies, real-time analytics, and ML. It gave birth to many customer demands like office automation, prior fault prediction of devices, and remote monitoring of applications. ML techniques open the potential for IoT applications by feeding information gathered by sensors into ML models, thereby applying results to enhance the business services [33]. Recommender system helps in fault prediction in smart office to predict faults at an early stage.

### 1.1. Motivation of Work

In this era, many people spend most of their time in offices or companies. The efficiency of employees is influenced by the environment of their workplace. To increase productivity, comfort is required in the office. So, the concept of the smart office is rapidly evolving and becoming the need of the hour. Smart office is a place where technology enables people to work properly, smartly, and speedily. It is a platform that enhances the capability of employees via different progressive technologies and tools. A smart office guarantees the active exploitation of IT resources and physical infrastructure. There is a need for predicting the faults in IoT-enabled devices to prevent devices from damaging. Thus, office automation allows the systems to become more transparent, which helps in achieving a decision that will result in the excellent functioning of an office. So, a smart office should be constructed to predict a fault early in any appliance [34].

### 1.2. Problem Statement

The study originates from the problem to automatically predict the fault in the office buildings. For offices that are big in size, it often becomes difficult to search for any faulty appliance in the whole office and to see if it needs replacement or not. The recommendation system is used to predict the fault in the office and the problems faced with the currently installed system are semiautonomous, no Internet connection, high cost, and the limited size of memory that stores user credentials. The problems mentioned above clearly depict that most of the recommendation systems are not user friendly and are not convenient to use for most of the users. A novel smart and autonomous recommendation system must be designed using machine learning techniques to provide an optimal solution.

### 1.3. Existing IoT Solutions in Smart Office

To enhance the performance of devices in a smart office, some existing solutions are suggested below [35]:

- *Business Assistants*. These virtual assistants synchronize with smart devices in the office to create an effective IoT environment. They have features of text-to-speech conversion, weather reports, meeting tracking, and many more.
- *IoT Tagging*. It is used for tracking the devices (i.e., monitor the current location or position of the device). These assets can be found out with the help of IoT tags.
- *Smart Thermostats*. They help in dynamically adjusting the temperature of the office, which makes the working environment more comfortable and cuts down the costs spent on inefficient control systems. They can be remotely controlled by voice assistance. They are used in buildings' HVAC to control different temperature zones.
- *Environment Monitoring Tools*. Some tools are required to monitor the devices in an office (i.e., whether they are working well or not).
- *Intelligent Lightning*. Smart bulbs can be used in offices that use the concept of motion sensors and adjust brightness and color balance throughout the day as per the user's requirement. It will also lead to less electricity bills.
- *Smart Printing*. A printer having an Internet connection monitors the paper as well as the ink of the printer and warns the person if it is getting low. It can also be connected to inventory systems to make orders for more actions without human involvement. Self-diagnostics in these smart printers are performed to notify the resource person about the quick fix or serious repair is required.
- *Smart Locks*. To keep offices safe and make entrance procedures easier for the employees, smart locks can be installed. These can be connected to attendance system to keep record of employee that when he is entering or leaving the office. Also, smart locks minimize the risk of break-ins.
- *Smart Meeting Room*. IoT is used to maintain a track of occupied meeting rooms as it is a must for every busy office.
- *Smart Vacuums*. Custodial staff is required to maintain cleanliness or pick up the slack, but they may cause a disruption to a security hole. An office can save from this by using a robotic vacuum and even they warn when they need to be emptied.
- *Smart Coffee Machines*. Coffee keeps up the productivity level of the employees. These machines keep the machine material in stock and keep a track of caffeine intake.

In this paper, a prototype of a smart office using IoT, cloud, and ML is designed that can control and automate devices at the workplace. The proposed architecture helps to forecast whether the device needs repairing or replacing when a fault a predicted. The major contributions of the paper are as follows:

1. The concept of fault prediction in IoT devices is elaborated where the role of ML in fault prediction to get accurate results is explained.
2. Furthermore, the use of the recommender system for fault prediction in the smart offices is discussed.
3. Also, the existing IoT solutions are described that enhance the performance of devices in the smart office.
4. An in-depth systematic literature survey is done to discuss the role of ML techniques in IoT devices.
5. An architecture is proposed that connects all office devices via IoT technology and uses a machine learning algorithm for fault prediction in IoT-enabled devices. Experimental setup, device specifications, and methodology of a new automated environment which is the integration of cloud, IoT, and ML are defined.

The rest of the paper is organized as follows. In Section 2, a related literature survey of the recent studies is carried out and based on that some conclusions have been derived.  Section 3 presents the proposed architecture of the work with its hardware specifications and experimental setup.  Section 4 highlights the methodology used to implement the proposed work.  Section 5 describes the workflow for fault prediction in office automation.  Section 6 concludes this study.

## 2. Literature Survey

In the present work, a comprehensive literature study has been carried out for fault prediction based on different ML techniques in IoT applications. Liu et al. [32] presented a framework of self-learning sensor fault detection that represented the sensor value, relationship, and status transformation. The group-based fault detection (GbFD) algorithm detected the fault in the sensor for validation in data of an oil field. The results showed that this method successfully detected 95% of total faults in the simulation data that carries around 752 million samples out of 5800 sensors. In addition to this, Vibhute and Gundale [36] presented a sensor failure prediction model. The sensor failure prediction involves the collection of sensor output data and the implementation of algorithms to anticipate impending failure. The algorithm represents the behavior of the system by identifying the factors contributing to sensor failure and then a predictive model is defined. This modeling is followed by the test data to check the reliability of the predictive model. With this implementation, the sensor failure with 98-99% accuracy was predicted as this prediction is applicable for all nonlinear systems. The proposed system has grown in accuracy and sensor maintenance can be done to fulfill reliability requirements. Early fault detection can minimize plant downtime, extended equipment life, increase safety and reduction in manufacturing costs.

For the very first time, Cicirelli et al. [37] proposed a meta-model of the smart environment. It exploits the concepts that are specific to the smart office application. A case study was presented by following the guidelines regarding its design and implementation. It helped in optimizing the architectural design. Then, Furdik et al. [38] presented a prototype of a smart office system which was developed as an application of the ELLIOT project. The described solution was based on the LinkSmart semantic middleware which is an open-source technology used for the development of IoT applications. They discussed principles of the system architecture and demonstrated on this prototype by using user experience monitoring approach and continuous evaluation was done on social and business parameters.

Xu et al. [39] systematically summarized the recent state-of-the-art industrial IoT. The paper reviewed the current researches of IoT in industries. The service-oriented architecture models of IoT were introduced and then basic technologies used in IoT were also discussed. Also, the essential applicability of IoT in industries was introduced. After that, the upcoming trends and research challenges linked with IoT were investigated. This paper focuses on the applications of IoT in industries and highlights the difficulties and potential possibilities for industrial researchers in the future. In addition to the previous, Mundada et al. [40] emphasize on the software fault prediction technique which is based on an artificial neural network with a back-propagation learning algorithm. Artificial Neural Network is adopted to locate the erroneous module and predict them. The results concluded that artificial neural network trained by utilizing resilient back-propagation produces better results rather than the algorithm of conventional back-propagation. Also, Barbosa et al. [41] presented a recommendation service named RS4IoT for smart devices. It provided an API that performs recommendation tasks for multiattribute sensors as informed by client applications which contain the features of sensors to be recommended. Also, RS4IoT helps users to evaluate some sensors and actuators after interacting in their social networks and gauges their importance in the recommendation.

Bakker et al. [42] studied the occupancy-based lighting control in an office affected by the potential of energy savings under different sizes of control zones. This strategy helps in optimizing the lighting control at room level as it can provide the first qualitative and quantitative advantages. The results concluded that it was beneficial to implement occupancy-based lighting in an office at each desk level. However, Rao et al. [43] focused on energy management in office cubicles and employee login information. A grid-based user interface is implemented to observe the occupancy of the employee in the office cubicle. A load cell and ultrasonic sensor are used to fetch the information of employee availability at designated cubicles. The fetched data is sent to the secured office cloud database through ESP8266 Node MCU for further control of the electrical appliances in office. The administrator can switch ON or OFF the required office electrical appliances.

With the advancement, Bhavana et al. [44] suggested a model that involves monitoring each home device through the Internet and detection of faults without human interference. The paper primarily emphasizes fault prediction in real-life devices. It uses the calculation of Naive Bayes for checking the abnormal condition in the devices. Hence, the proposed system helps in fault detection and saves time. Cloud computing, IoT, and mobile app are used in the implementation of this proposed solution; that is why it is called a multitechnology environment as many technologies are used in the system. Arun et al. [45] presented a smart office system based upon the IoT application. The smart office contains the biometric for opening the door locks, temperature and humidity sensor, smoke detection sensor for fire indication, and automatic lighting system. The fingerprint biometric sensor was used for security purposes so that other people cannot arrive at the office area. When any unauthorized person enters the office area, the buzzer will ring in control room and an e-mail will be forwarded to security guards. In this system, there were two working modes: one is automatic mode, and another is manual mode.

In 2018, Gouthaman and Suresh [46] emphasized on risk analysis and management of the development of agile software using IoT and cloud computing. The authors proposed a framework that includes a design of IoT-Fog-based agile software risk management as well as an assessment system. They focused on different types of risk in the IoT-Fog-based frameworks that could end up being more effective. The fundamental goal was to address the significance of the agile approach and the importance of risk management towards cutting edge frameworks such as cloud, Fog, and IoT utilizing relevant tools. Whereas, in 2020, Bak et al. [47] proposed an approach that visualizes applications of IoT as a collection of IoT services. They proposed an event-flow-based visualization technique where an IoT service is viewed as a flow from event to action. A tool named SmartVisual was implemented by the authors that perform a static investigation on SmartApps to create an event flow diagram. This tool assesses the inputs, actions, events, and event flows of 64 samples of SmartApps which are rendered by SmartThings. Each SmartApp had 2 input devices, 2 output devices, and 4 event flows. In 2019, Xenakis et al. [48] presented an IoT and cloud-based framework for fault prediction and machine condition monitoring for Industrial IoT. This study provided real-time cloud-oriented maintenance using the tool MATLAB. To minimize the cost, the authors founded a cross-layer optimization problem for adequate energy consumption using a method of multipliers algorithms.

Bhatnagar et al. [29] summarized different ML techniques that proved to give better results and improve speed for prediction and classification. These technique improves the various performance parameters of the system like the reduction of noise, recovered lost data, increase prediction rate (using device location and state) to achieve better and faster results. The error reduction rate is approx 1% using clustering algorithms, neural networks, and Bayesian network. Other techniques like decision trees, regression analysis, Principal Component Analysis, *k*-nearest neighbors algorithm, random forests, genetic algorithms, and support vector machines also give great results. The ML algorithms predict the changes themselves due to their learning properties. ML algorithms tend to decide to achieve a goal. Thus, it is clear from the above that the ML algorithms decrease the error rate in IoT. Also, Souri et al. [49] presented a prediction model with particle swarm optimization and multilayer perceptron for formal verification and behavioral modeling using ML. Also, the defect metrics were detected for the verification of the fault prediction behavior in IoT applications. It is observed from the result that the verification method has very little operating time and memory usage as compared to other methods. However, Lo et al. [50] summarized the various approaches that are used to diagnose the industrial complex system using artificial intelligence. The articles published from 2002 to 2018 were covered for fault diagnosis using ML tools in industrial systems. In addition to this, Pathak et al. [51] developed an IoT-based system that is used to monitor the patient's position without a hidden activity. The basic target of this system is to monitor the patients' subtleties. The system was built to enhance speed and accuracy rate. Data is analyzed based on age, time, obesity, month, heartbeat, and temperature and humidity using *R* and implemented the use of linear regression and decision tree for analyzing the accuracy. The authors discussed about the IoT-based recommendation technologies that will recommend future IoT solutions. [52].

Meena et al. [53] proposed a system that localizes a person and controls the devices. An indoor localization technique was applied to localize a person. This technique obtains the location of an individual inside a room using RFID tags and PIR sensors by identifying their patterns. After the implementation of the system, the authors prove that energy consumption was comparatively less. Also, Jia et al. [54] investigated the recent projects and technologies of IoT used for smart building development in academia and industry contexts. Afterward, they selected some latest IoT building applications to build smart buildings. They also discussed some challenges and future research questions on IoT integration in smart buildings. They concluded that there is a need for more work from researchers in this field.

Nan [55] introduces a process that designs and implements a network monitoring system using VC++ platform to monitor network traffic and detect suspicious data while accessing database records to achieve network security. Whereas Wang et al. [56] propose a collaborative office automation system that improves the work efficiency of team. This system has feature of continuous and stable operation that saves resources.

After reviewing the above discussed literature survey and 1651 papers from the Scopus database, the following conclusions have been derived:

- In the last 10 years from 2012 to 2021, the number of papers published is increasing year by year as shown in Figure 4. The maximum number of papers is published in 2019 and the annual growth rate is 5.5%.
- 3-Field plot applies clustering technique that correlates different parameters like keyword, country, and year.  Figure 5 shows in which year, how the different countries use multiple keywords. In the year 2015, this work gained an increase and USA, China, and India are the leading countries.
- In Figure 6, the top five sources in which maximum papers published are shown. This figure represents the documents published in specific sources year-wise. The maximum papers, i.e., 31, are published in ACM International Conference Proceeding Series followed by Advances in Intelligent Systems and Computing having 22 papers. Constant growth is seen in the IEEE Internet of Things Journal.
- Figure 7 shows the trending topics as per the author keywords year-wise. Each keyword has a minimum frequency of 15 and the anomaly detection, sensors, deep learning are the latest keywords.

## 3. Proposed Framework for Office Automation

IoT-based appliances enhance the performance of the system and reduce human intervention. The proposed architecture performs all the tasks automatically while interacting securely with appliances. The main focus of this proposed architecture is to connect all office appliances using the Internet with the help of IoT technology. The novelty of this work is to develop a smart and autonomous recommendation system for prediction of faults using a machine learning technique.  Figure 8 is the proposed fault prediction system using an ML algorithm. It contains electrical office appliances, sensors, and a database server. It has a live monitoring feature on the cloud that can be accessed by users and an ML-based fault prediction algorithm that predicts faults in the appliances. Cloud has features of nonvolatile memory and excess space, so the data can be retrieved from it on regular basis. When office appliances are ON, then this system starts checking the health of appliances and in case of any abnormal values, the fault prediction mechanism starts. A primary unit of the proposed architecture is the ML algorithm. The ML algorithm predicts the inevitable faults based on the analysis of the existing dataset and also, divides or clusters the obtained data based on similarity. This collected data is stored on the cloud so that this data can be used for fault prediction in IoT-enabled appliances in the future. Also, this algorithm finds the similarity among different datasets based on prior data available with the algorithm. This work is implemented in the IoT-enabled office to predict both healthy and unhealthy appliances.

A software application keeps the track of live monitoring of cloud data received from appliances. Hence, if any appliance does not work in normal conditions, then the fault can be predicted and matched with the existing fault by ML algorithm and a relevant solution will be recommended. Also, an alert message will be delivered on the concerned person's smartphone when any abnormal functioning of the appliance is predicted. The data fetched is utilized by the ML algorithm to determine faults that are going to happen or had already occurred. This is the pivotal functionality of the proposed architecture. The end-user can monitor the power consumption of each and every office appliance and determine the future prediction of any fault. Any change in observed values sends an alert message to the end-user. Hence, the proposed architecture will predict the fault at an early stage and prevents the damage of the appliance.

### 3.1. Experimental Setup

The proposed architecture consists of an ATmega8 microcontroller that works as the fundamental controller. This framework deals with continuous real-time monitoring of the electrical appliances through current sensors that can be remotely controlled. The inputs from different sensors are checked against the constant gadget working. A gas sensor is used to detect toxic gases or identify any gas leakage whereas the temperature and humidity sensor is used to control air conditions. An ultrasonic sensor is used to detect object proximity.  Figure 9 presents the block diagram of smart office.

Figure 10 shows the prototype of the smart office which controls the appliances in office by the occupancy and movement of office staff. This paper represents the implementation of a new system for office employees to control electric appliances automatically and save energy. This framework is better than other existing frameworks because of the following:

- The office is monitored unit-wise rather than exercising the whole office space
- It is economical and cost-efficient as an ATmega8 microcontroller is deployed
- A 16 × 2 LCD is used to check the status of appliances as well as the security of the office
- The WiFi module is used to send an alert message to the end-user

### 3.2. Hardware Components

- *ATmega8 Microcontroller*. ATmega8 microcontroller is the cheapest microcontroller and provides many features in lesser pins. It consists of 1 kilobyte of SRAM and 512 bytes of EEPROM. The ATmega8 application is very versatile because of the program memory of 8 kilobytes. Due to its compact size, it can be placed on many small boards.
- *WiFi Module*. ESP8266 WiFi module is used for endpoint IoT developments. It has an integrated TCP/IP protocol stack and can be controlled from a local WiFi network. ESP8266 has low cost and high functionality, which makes it an ideal module for IoT. It fetches data from the Internet using API's and accesses any information available on Internet, thus making it smarter.
- *Current Sensors*. ACS712 current sensor is applied to measure the current flowing within a wire. It uses the concept of the magnetic field to sense the current and produce a proportional output. It is used with both AC and DC. It determines energy usage and keeps the cost down to increase efficiency. They help in predicting faults in a device and prevent damaging of equipment.
- *Gas Sensor*. MQ-135 gas sensor is applied in air quality control equipment to measure common air quality gases such as CO_2_, smoke, NH_3_, NO_x_, alcohol, and benzene. The detection range of this sensor is 10∼1000 ppm. It detects different types of toxic gases and is known as a low-cost sensor for such kinds of applications. It is ideally used in offices with a monitoring circuit.
- *Temperature and Humidity Sensor*. DHT11 sensor calculates humidity from 20 to 90% and temperature from 0°C to 50°C with an accuracy of ±1% and ±1°C, respectively. It is an economic digital sensor that employs a thermistor and capacitive humidity sensor to estimate the surrounding air. It can be easily interfaced with the ATmega8 microcontroller.
- *Ultrasonic Sensor*. SR04 ultrasonic motion detection sensor is applied to detect the motion of moving objects. It is used in automatic door opening devices and contact-less-speed measurement equipment. They are also able to measure an approaching or receding object.
- *Power Supply*. Any IoT device will need electricity to work whether it comes from a power outlet or a battery. A certain amount of voltage and current is always required.
- *16 × 2 LCD Screen*. In this, 16 × 2 indicates two lines per column and each line has 16 columns, so a total of 32 characters. To display custom text, numbers, and special characters, it is programmed using a microcontroller board with the liquid crystal library.

## 4. Proposed Methodology

This section defines a methodology of a new automated environment which is the integration of cloud, IoT, and ML. In the literature survey section, many researchers separately research in one domain taking into consideration their unique properties, features, attributes, advantages, and disadvantages. But the proposed architecture features all these concepts and finds a new way to integrate them into a new concept by analyzing their common features. Faults are predicted in IoT appliances to enhance their performance and reliability. The existing fault dataset and device's current status are maintained to observe changes in values which could lead to a fault that can be prevented at an early stage. The proposed architecture fetches data from office appliances to enhance the performance of each appliance. The data being collected by IoT is sent to the ML algorithm for future fault prediction. This data stored in database is connected to a cloud server. The prediction and classification process of faults is done via an ML algorithm. Then, this information is shared with the end-user as well as the solutions will be recommended using a mobile application. The mobile application with the end-user comprises software that keeps track of all devices and alerts the user on deviation or abnormal functioning of any appliance.

## 5. Workflow for Fault Prediction in Office Automation

Figure 11 shows the analysis of the flow of the faults. Initially, data from all IoT appliances in a smart office like electrical appliances or sensors is gathered. This gathered data is saved on a server that is responsible for controlling all the IoT devices. Then, this data is being preprocessed for fault identification and prediction. Once the faults are identified, then they are analyzed through ML. Also for excess data, the smart office server transfers data to the cloud and users can remotely access all data via a software application interface on their smartphone. The solutions will be recommended for identified faults. An Internet connection allows the user to communicate with the smart office to get all the details and remotely handle devices if that person is not in the office.

A complete flowchart of our proposed architecture is shown in Figure 12. The working model of our proposed architecture firstly requires initializing all devices and sensors in the smart office. Then, the data fetched from all devices is preprocessed using ML. Then, the status of each and every device is checked. Every device will have 2 states, either healthy or unhealthy. If the device is in a healthy state, then normal working will take place. If the device is in an unhealthy state, then the fault prediction and classification process will take place. The solutions will be recommended whether the device needs repairing or replacing, and a notification will be sent to the concerned person's smartphone and an e-mail will be sent to the guard who will repair the fault or replace the device.

## 6. Conclusion

Machine learning is a growing technology that plays a vital role in the advancement of the IT sector. The proposed architecture presents a prototype of a smart office that uses IoT, cloud, and ML technology for office people so that their efficiency can be increased. It has a multitechnology environment as many technologies are involved in this. Live monitoring of office appliances helps in the early fault prediction without any intervention of human effort and also saves the maximum power of office appliances. This proposed architecture identifies and classifies the faults before their occurrence and hence, recommends the most suitable solution that can be used for fixing these faults in a smart office. ATmega8 microcontroller is used to automatically control the devices present in the smart office. The current sensors, temperature and humidity sensors, detection sensors, and gas sensors are being premeditated in this system to make the work more relaxed. Whenever the values are not normal, a notification will be flashed on the end-user smartphone and an e-mail will be forwarded to the concerned security person. The smart office system is prolonged to the whole smart building. The fault prediction capabilities can be expanded to include fault diagnosis, identification, and prognosis. This paper proposed a solution to manage and monitor the office cubicles easily. This proposed system provides many advantages like security, improved comfort, and saves energy and cost. Thus, it helps to build an autonomous environment in a smart office. In the future, new technologies and techniques could be investigated to enhance the performance and reliability of IoT appliances.

## Figures and Tables

**Figure 1:** Architecture of an IoT application [3–6].

**Figure 2:** IoT and its application areas [11–13].

**Figure 3:** Integration of IoT with cloud [21–23].

**Figure 4:** Number of documents published year-wise.

**Figure 5:** 3-Field plot classification of published papers by year, country, and keyword.

**Figure 6:** Number of documents per year per source.

**Figure 7:** Trending topics as per the author keywords.

**Figure 8:** Framework for office automation.

**Figure 9:** Block diagram of smart office.

**Figure 10:** Prototype of the smart office.

**Figure 11:** Analysis of fault flow diagram.

**Figure 12:** Flowchart of the proposed architecture.

## Data Availability

The data used to support the findings of this study are available from the corresponding author upon request (gdhiman0001@gmail.com).
